# Baicalin Alleviates Thrombin-Induced Inflammation in Vascular Smooth Muscle Cells

**DOI:** 10.1155/2022/5799308

**Published:** 2022-01-21

**Authors:** Xiaolei Zheng, Ping Wang, Mengqi Jia, Qing Li, Anna Zhang, Qingbo Zhou

**Affiliations:** ^1^Department of Neurology, the Second Hospital, Cheeloo College of Medicine, Shandong University, Jinan 250033, China; ^2^Institute of Medical Sciences, the Second Hospital, Cheeloo College of Medicine, Shandong University, Jinan 250033, China; ^3^Department of Geriatrics, South Branch of the Second Hospital, Cheeloo College of Medicine, Shandong University, Jinan 250000, China; ^4^School of Nursing and Rehabilitation, Cheeloo College of Medicine, Shandong University, Jinan 250012, China

## Abstract

Atherosclerosis (AS) is a chronic inflammatory disease of the arterial intima. As AS represents the most common type of vascular disease, it affects millions of individuals and is a source of high morbidity and mortality rates worldwide. Overwhelming evidence indicates that AS-related inflammation is mediated by proinflammatory cytokines, chemokines, adhesion molecules and inflammatory signaling pathways, with each of these factors being shown to play critical roles during the entire progression of AS. While a number of drugs have been approved for use in the treatment of AS, their benefits are modest, which underscores the urgency for the development of new drug therapies. In part, these deficits in effective drugs can be attributable to the lack of a clear understanding of the molecular mechanisms of AS. In this study, we investigate the capacity for thrombin to trigger inflammation and induce cell proliferation in vascular smooth muscle cells (VSMCs). We then assessed the effects of baicalin and its potential mechanisms on VSMC inflammation as induced by thrombin. Baicalin, which is a natural bioactive compound of S. baicalensis Georgi (SBG), exerted a protective effect against thrombin-induced VSMC inflammation as resulting from the upregulation of PAR-1. This protection as exerted by baicalin appears to reside in its capacity to produce an inhibitory effect on the thrombin-induced activation of the ERK1/2 pathway. These findings suggest that baicalin may be a promising candidate for the treatment of atherosclerosis.

## 1. Introduction

Arteriosclerosis (AS), one of the most common types of vascular disease, has become the focus of extensive basic and clinical research due to the serious nature of its effects upon cardiovascular and cerebrovascular diseases [1]. Overwhelming evidence has accrued indicating that AS is a chronic inflammatory disease, involving different cell types, multiple cytokines and adhesion molecules [2]. The proliferation of vascular smooth muscle cells (VSMCs) represents a critical event in the development of AS [3]. And, Kalz et al. have recently proposed that thrombin, as a component of the coagulation-inflammation axis, is a key factor in regulating the inflammatory processes of AS [4].

Thrombin is a procoagulant and proinflammatory serine protease [5]. It acts as a powerful modulator of many processes involving regulation of permeability, migration and proliferation of VSMCs, induction of multiple pro-inflammatory markers and recruitment of monocytes into the vascular lesions, all of which are related to the progression of AS [6, 7]. Unlike its activity within the coagulation cascade, its cellular pro-inflammatory and proatherogenic effects are primarily mediated by the protease activated receptor 1(PAR-1) in humans [8]. Protease activated receptors (PARs), a small family of G protein-coupled receptors (GPCR), are comprised of four members (PAR-1, 2, 3 and 4) and normally show low levels of expression within contractile VSMCs. However, under conditions related to endothelial dysfunction, expressions of PARs are significantly up-regulated [9]. This thrombin-PARs interaction triggers several mechanisms including, increasing the expression of cell adhesion molecules, inducing the secretion of pro-inflammatory cytokines, activating inflammatory responses of atherosclerotic plaques, stimulating VSMCs proliferation and aggravating vascular lesions at injury sites. As all of these factors can contribute to the pathology of AS, inhibition of this thrombin-PAR interaction has been identified as a potentially important target for the treatment of AS [5, 10]. In fact, results from recent studies have indicated that novel thrombin inhibitors show significant therapeutic potency in the treatment of AS through their ability to inhibit inflammatory responses [11].

A substantial amount of evidence has been presented suggesting that AS is a chronic inflammatory disease of the arterial intima and involves proinflammatory cytokines, chemokines, adhesion molecules and inflammatory signaling pathways [12]. Proinflammatory cytokines including IL-1*β*, IL-6 and TNF-*α* have all been shown to play a vital role in AS-related inflammation. Therefore, inhibiting the production of these cytokines may prove beneficial in the anti-inflammatory treatment of AS. Compared with unaffected tissue, the expression of IL-1*β* in atherosclerotic lesions is elevated, suggesting that IL-1*β* may serve as a potential clinical target for the anti-inflammatory treatment of AS [13, 14]. NF-*κ*B is the main regulator of inflammation and immune homeostasis that can be induced by gene encoding, proinflammatory cytokines, chemokines, adhesion molecules and monocytes bound to the endothelium. Accordingly, it plays a central role in inflammatory diseases and other diseases with significant inflammatory components, such as rheumatoid arthritis, cancer and atherosclerosis [15, 16]. In mammals, the NF-*κ*B/Rel family is comprised of p50, p52, p65 (Rel-A), c-Rel, and Rel-B proteins. These proteins usually form homo- or hetero-dimers and combine with NF-*κ*B inhibitor (I-*κ*B) proteins to remain in an inactive state in resting cells [17]. The richest form of NF-*κ*B, as activated by pathologic stimuli via the canonical pathway, is the p65: p50 heterodimer. A disproportionate increase in activated p65 and subsequent transactivation of effector molecules are indispensable for the pathogenesis of numerous chronic diseases including AS [18, 19]. Li et al. demonstrated that microRNA-145 accelerated inflammation in atherosclerotic cells and mice by activating NF-*κ*B signaling [20]. In addition, Zhang et al. reported that in a rat model, FGF-21 significantly downregulated the levels of Rho kinase and NF-*κ*B, which helped alleviate AS [21].

Several signaling pathways regulate the pathogenic process of AS, including inflammatory processes, endothelial cell activation, monocyte/macrophage recruitment and activation and smooth muscle cell proliferation, with MAPK pathways playing a key role [22, 23]. MAPKs, a group of serine or threonine protein kinases conserved in eukaryotic species, are essential for the development, differentiation, learning, memory, and secretion of paracrine and autocrine factors [24]. Of the three well-defined MAPK pathways identified (i.e., the ERK1/2, JNK and p38 kinase pathways) [25], ERK1/2 kinase is involved in thrombin-stimulated VSMC proliferation [26], and thus plays a vital role in the inflammatory process of AS [27]. Li et al. showed that imperatorin reduces the inflammatory response of AS by regulating MAPKs signaling as demonstrated in both in vivo and in vitro models [28]. In the past decade, an eruption of new studies has provided valuable insights into ERK1/2-NF-*κ*B pathways, which have greatly contributed to our understanding of diseases such as AS [29, 30]. Pan et al. reported that LncRNA H19 promoted AS by regulating MAPK and NF-*κ*B signaling pathways [31]. Interestingly, work within our laboratory has revealed that baicalin, the main bioactive ingredient of Scutellaria radix, inhibited activation of the NF-*κ*B p65 and ERK1/2 signaling pathways in thrombin-induced human umbilical vein endothelial cells (HUVECs). This capacity for protecting cells from damage laid the foundation for further investigations into the anti-atherosclerotic mechanisms of baicalin in VSMCs.

Baicalin has served as a Traditional Chinese Medicine for thousands of years. Experimental and clinical evidence indicates that the flavonoid baicalin exerts various pharmacological activities, including anti-oxidant, anti-inflammatory, anti-apoptotic and anti-excitatory effects [32]. In particular, its anti-inflammatory effects have been confirmed in a variety of disease models, including diabetes [33], cardiovascular diseases [34], cerebrovascular and neurological disorders [35], and carcinogenesis [36]. According to results from a number of reports, its anti-inflammatory effects mainly involve attenuating the activity of NF-*κ*B and suppressing the expression of some inflammatory cytokines and chemokines (i.e., monocyte chemotactic protein-1 (MCP-1), cyclooxygenases, tumor necrosis factor (TNF) and interleukins (IL)) [37, 38]. Previous results from our laboratory have demonstrated that baicalin had a protective effect on thrombin-induced cell injuries in HUVECs, and the potential anti-inflammatory mechanisms of baicalin may involve an inhibition of thrombin-induced NF-*κ*B activation and PAR-1 expression [39]. However, whether baicalin has a protective effect on thrombin-induced inflammation in AS remains unknown.

In this study, we treated VSMCs with thrombin to induce the inflammation that occurs in AS and assessed the involvement of PAR-1 protein in this process. In addition, the effects of baicalin and its underlying mechanisms within this thrombin-induced inflammation model were then investigated.

## 2. Materials and Methods

### 2.1. Reagents, Chemicals and Antibodies

Thrombin (T6884), dimethyl sulfoxide (DMSO; D5879) and baicalin (CAS Number: 21967-41-9; purity, 98%; molecular formula, C21H18O11; molecular weight, 446.36) were purchased from Sigma-Aldrich (St. Louis, MO, USA); Fetal bovine serum (FBS; 10099-141) from Gibco; RPMI-1640 (SH30809.01B) from Hyclone; Cell Counting Kit-8 (CCK-8; C0038) from Beyotime. PrimeScript™ RT reagent Kit and TB Green® Premix Ex Taq from Takara (Dalian, China). PAR-1 (A5641) antibody from Abclonal. NF-*κ*B (8242), p-P65 (3033), ERK1/2 (4695), p-ERK1/2 (4370) antibodies were from Cell Signaling Technology (CST). ACTB (66009-1-Ig) antibody was from Proteintech. Goat anti-rabbit IgG antibody (5220-0338) from seracare.

### 2.2. Cell Lines, Cell Culture and Drug Treatment

Rat aorta vascular smooth muscle cells (RA-VSMCs) were purchased from the American Type Culture Collection (ATCC, Manassas, VA, USA). Cells were cultured in RPMI-1640 supplemented with 10% fetal bovine serum (FBS, Gibco), penicillinG (100 U/mL), and streptomycin (100/mL) in a 5% CO2 incubator at 37° C. Cells of the 4-8 generation were employed in all experiments. In experiments for thrombin stimulation, cells at 60–70% confluence were pretreated with baicalin at different concentrations (0, 10, 20 or 50 uM) for 2 hours, followed by treatment with thrombin (2.5 U/mL) for an additional 24 hours.

### 2.3. Cell Proliferation Assay

Cells were seeded in 96-well plates at a density of 5 × 10^3^ cells per well and cultured for 24 hours. Cells were then treated with compounds at the indicated concentrations for specific times. After drug treatment, cell proliferation was measured with use of the CCK-8 assay [40]. Briefly, 10 *μ*l CCK-8 solution (5 mg/mL) was added into each well of 96-well plates, followed by further incubation of 2 hours at 37° C. Absorbance was then determined at a wavelength of 450 nm with a microplate reader (BioTek, CYTATION5MF, USA). All experiments were repeated 3 times.

### 2.4. Immunocytochemistry

Immunocytochemical staining was performed as described previously [41]. Briefly, cells were seeded on cover slips overnight. After drug treatments, cells were fixed in 4% paraformaldehyde for 30 min followed by incubation with the primary antibody (antiPAR-1) overnight at 4°C. After washing with PBS, cells were incubated with PE-labeled secondary antibodies (1 : 500; Invitrogen) for 1 hour at room temperature and then counterstained with 4–6-diamidino-2-phenylindole (DAPI) for 10 minutes. Images were obtained with use of laser scanning microscopy (NIKON ECLIPSE 90i, LH-M100CB-1, Japan).

### 2.5. RNA Extraction and Quantitative Real-Time Polymerase Chain Reaction

Total RNA was extracted from VSMCs with use of Trizol RNA-RNAiso Plus. Reverse transcription was conducted to generate complementary DNA (cDNA) using the Prime Script RT reagent kit with gDNA Eraser according to manufacturer's protocol. The mRNA expression of IL-1PAR-1 was determined by quantitative real-time PCR using SYBR premix Ex Tap TM (TLiRNSEHPLUS). Predesigned primers were as follows: *β*-actin: 5'-CTCTGTGTGGATTGGTGGCT-3' (forward primer), 5'-CGCAGCTCAGTAACAGTCCG-3' (reverse primer); PAR-1: 5'-GCCACCGCAGCGTTTTATTG-3' (forward primer) and 5'-CAGGTGGTGATGTTGAGCCC-3' (reverse primer); IL-1*β*: (forward primer) 5'- AAGCAGCTATGGCAACTGTCC-3' and (reverse primer) 5'- TCATCTGGACAGCCCAAGTCA-3'. *β*-Actin was used as internal control. Finally, relative mRNA expressions of these genes were calculated using the 2(−*ΔΔ*Ct) method.

### 2.6. Western Blotting

After treatment, cells were collected and gently washed twice with PBS. Total proteins were extracted from cells using protein lysis buffer (1% SDS in 25 mM Tris-HCl, pH 7.5, 4 mM EDTA, 100 mM NaCl, 1 mM PMSF, 1% cocktail protease inhibitor). Samples were centrifuged at 12,000 g for 15 min at 4°C and supernatants collected. Protein concentrations were determined using the Coomassie brilliant blue protein assay. Equal amounts of protein (50 mg) were resolved by SDS-PAGE, and then transferred onto nitrocellulose membranes. After being blocked with 5% non-fat dry milk in TBS for 1 h at room temperature, membranes were incubated with primary antibodies (1 : 1000) overnight at 4°C. After washing, membranes were treated with appropriate secondary antibodies for 1 h at room temperature. Finally, immunocomplexes were detected with an enhanced chemiluminescence plus kit.

### 2.7. Statistical Analysis

All statistical analyses were performed using SPSS 19.0 software. All data were presented as means ± Standard Error of Mean (SEM). Differences between groups were evaluated using a two-tailed Student's t test or for greater than two groups using one-way ANOVA with multiple comparisons. A value of p <0.05 was required for results to be considered as statistically significant.

## 3. Results

### 3.1. Thrombin Induces Proliferation of VSMCs

An increasing body of evidence has been presented suggesting that thrombin plays a critical role in promoting the proliferation of VSMCs, thereby contributing to the pathogenesis of AS [42, 43]. To assess the effects of thrombin on VSMC viability, an CCK-8 assay was used. Cell viability was significantly increased after exposure to 1, 2.5 or 5 U/ml thrombin for 24 h, while cell proliferation was induced by 2.5 U/ml thrombin at 24, 36 and 48 h after treatment (Figures 1(a) and 1(b)). Thus, thrombin induced the proliferation of VSMCs in a dose- and time-dependent manner.

### 3.2. Thrombin Induces Inflammation in VSMCs

According to reports, thrombin is involved in inflammatory processes contributing to AS in VSMCs. These effects involve a critical role for the transcription factor NF-*κ*B, as well as an involvement of IL-1*β* [10]. In this study, we evaluated the effects of thrombin on VSMC inflammation by monitoring the expression of IL-1*β* mRNA and activation of NF-*κ*B (P65) protein, as measured by determining phosphorylated P65 protein levels. RT-PCR was used to determine levels of IL-1*β* mRNA, while Western blotting was used to detect phosphorylated NF-*κ*B (P65) protein. After exposure to thrombin (1, 2.5 or 5 U/ml), levels of IL-1*β* mRNA (Figure 2(a)) and phosphorylated NF-*κ*B (p-P65) (Figure 2(b)) in VSMCs were increased in a dose-dependent manner. These data indicate that thrombin induced inflammation within VSMCs in a dose-dependent manner.

### 3.3. Thrombin Induces Upregulation of PAR-1 in VSMCs

Results from a number of studies have indicated that the cellular actions of thrombin in the pathogenesis of AS are mediated by the upregulation of protease-activated receptors (PARs) [9]. Accordingly, we tested whether thrombin could induce an upregulation of PAR-1 in VSMCs. After exposure to thrombin (1, 2.5 or 5 U/ml), levels of PAR-1 mRNA and protein in VSMCs increased in a dose-dependent manner (Figures 3(a) and 3(b)). These results indicate that thrombin induced an upregulation of PAR-1 in VSMCs.

### 3.4. Baicalin Inhibits Thrombin-Induced Proliferation of VSMCs

Experimental and clinical studies have shown that baicalin is an active flavonoid compound with a variety of pharmacological activities, including anti-oxidation, anti-inflammatory, anti-apoptosis and anti-excitotoxicity [32]. Here, we used a CCK-8 assay to investigate the effects of baicalin on the proliferation of VSMCs as induced by thrombin. Treatment with 2.5 U/ml thrombin for 24 h increased cell viability by approximately 1.3-fold of that obtained with untreated control cells (Figure 4(a)). However, pretreatment with baicalin (10, 20 or 50 *μ*M) reduced the viability of these VSMCs as induced by thrombin (Figure 4(a)). Moreover, as shown in Figure 4(b), cell viability did not decrease after exposure to any of these concentrations of baicalin (10, 20, 50 *μ*M), which demonstrates a wide safety margin for this drug. These results indicate that baicalin inhibited the proliferation of VSMCs as induced by thrombin.

### 3.5. Baicalin Alleviates Thrombin-Induced Inflammation in VSMCs

Our previous findings have revealed that activation of NF-*κ*B and upregulation of IL-1*β* mRNA in VSMC inflammation, as induced by thrombin, contributes to the progression of AS. Here, we investigated the effect of baicalin on the activation of NF-*κ*B and upregulation of IL-1*β*, as induced by thrombin, in VSMCs. Expression levels of IL-1*β* mRNA were determined using RT-PCR, while NF-*κ*B (P65) and p-P65 protein levels determined with Western blotting. As shown in Figures 5(a) and 5(b), compared with control cells, the expression of IL-1*β* mRNA and level of p-P65 protein in VSMCs treated with 2.5 U/ml thrombin increased significantly, while administration of baicalin (10, 20 or 50 *μ*M) attenuated this upregulation of IL-1*β* mRNA and p-P65 protein in a dose-dependent manner. Thus, baicalin alleviated thrombin-induced inflammation in VSMCs.

### 3.6. Baicalin Inhibits VSMC Inflammation by Suppressing Thrombin-Induced PAR-1 Expression

Since thrombin has been identified as a serine protease that activates PAR-1 to trigger intracellular signaling pathways promoting cell inflammation, we investigated the effect of baicalin on the upregulation of PAR-1 in thrombin-induced VSMC inflammation. Levels of PAR-1 mRNA and protein were determined using RT-PCR and Western blotting, respectively. As shown in Figures 6(a) and 6(b), after 2.5 U/ml thrombin treatment, levels of PAR-1 mRNA and protein in VSMCs were significantly increased, an effect which was partially inhibited with an administration of baicalin (10, 20 or 50 *μ*M) in a dose-dependent manner. To visualize PAR-1 distribution, the PAR-1 protein was measured by immunocytochemistry using a PAR-1-specific antibody (Figure 6(c)).

### 3.7. The Inhibitory Effect of Baicalin on VSMC Inflammation Induced by Thrombin-PAR-1 Is Mediated via ERK1/2 Signaling

In recent years, several signaling pathways have been identified as being involved in the atherosclerotic inflammatory process through the thrombin-induced upregulation of PAR-1 in VSMCs, of which the ERK1/2 pathway plays a key role [23]. Therefore, we determined the phosphorylation of ERK1/2, a MAPKs subfamily, as a means of assessing the signaling pathways that mediate VSMC inflammation induced by thrombin-PAR-1. Thrombin treatment (1, 2.5 or 5 U/ml) increased the phosphorylation of ERK1/2 in a dose-dependent manner (Figure 7(a)). This increase in ERK1/2 phosphorylation as induced by thrombin (2.5 U/ml) was attenuated with the administration of baicalin (10, 20 or 50 *μ*M) (Figure 7(b)). Therefore, the inhibition of VSMC inflammation by baicalin, as induced with thrombin-PAR-1, appears to, at least in part, involve the ERK1/2 signaling pathway.

## 4. Discussion

AS is the principal pathological basis for cardiovascular and cerebrovascular diseases that eventually leads to high rates of morbidity and mortality worldwide. These issues emphasize the urgency for the development of new drug therapies directed at AS [1]. In this study, we provide the first evidence for a possible new drug in the treatment of AS. In specific, we show that baicalin can markedly inhibit thrombin-induced inflammation in VSMCs, as achieved by reducing the thrombin-induced upregulation of IL-1*β* mRNA expression and increase of phosphorylated NF-*κ*B (P65) protein. A possible mechanism for this effect of baicalin may involve an inhibition in the thrombin-induced activation of ERK1/2 signaling in VSMCs, thereby inhibiting VSMC inflammation mediated by thrombin-induced upregulation of PAR-1in AS. In short, our findings reveal a protective effect of baicalin on VSMCs inflammation and provide a potential strategy for the application of baicalin as an atherosclerotic therapy.

Increasing evidence has accrued which suggests that AS is a chronic inflammatory disease of the arterial intima [44]. AS-related inflammation, as mediated by proinflammatory cytokines including IL-1*β*, IL-6, TNF-*α*, chemokines, adhesion molecules and inflammatory signaling pathways, plays an important role in the entire atherosclerotic process [12]. Production of proinflammatory cytokines and chemokines induces the activation of NF-*κ*B that serves as a master regulator of inflammation, then promotes the progression of AS [45, 46]. In our study, we observed that VSMCs exposed to thrombin show an increase in the expression of IL-1*β* mRNA and phosphorylation of NF-*κ*B (P65) protein, thereby inducing the inflammatory process in AS. Notably, thrombin is a pivotal contributor to vascular pathophysiology. The cellular effects of thrombin on inflammation in AS are mediated by protease-activated receptors (PARs), which possess their own cryptic ligand that is unmasked by proteolytic cleavage [7]. Results from previous studies have indicated that an upregulation of PARs in VSMCs seems to be a key element in the pathogenesis of AS and contributes to the pro-inflammatory phenotype observed in endothelial dysfunction [47]. Our current findings demonstrate that thrombin induces an upregulation of PAR-1 mRNA and protein in VSMCs, which may then contribute to the inflammatory process of AS.

There also exists considerable evidence that VSMC proliferation is involved in the initiation and progression of AS. In the walls of normal blood vessels, VSMCs show low levels of turnover with minimal proliferation. However, in response to vascular injury, aberrant VSMC proliferation is observed which promotes the formation of atherosclerotic plaques [27, 48]. One example of vascular injury is that of thrombin, which stimulates VSMC proliferation and plays a key role in the inflammatory pathogenesis of AS [27]. Consistent with findings of previous studies, we observed an inductive effect of thrombin on VSMC proliferation as associated with increased cell viability in our study.

Despite the identification and attempts at treatment for AS that have persisted for over 100 years, it remains a condition that continues to affect millions of individuals, mostly presenting as myocardial infarctions, strokes and disabling peripheral artery disease. While numerous drugs have been approved for the clinical treatment of AS, their benefits are relatively modest [1]. Therefore, a great need exists for the development of more effective anti-atherosclerotic drugs. As a considerable amount of research has been directed toward investigating the pathogenesis of AS, the focus of drug development has shifted to strategies involved with reducing the inflammatory pathogenicity associated with this condition [34]. Increasing evidence of late has indicated that augmented inflammation in AS is harmful, suggesting that suppression of this inflammation in AS may prove to be an effective therapy. Li et al. reported that cinnamaldehyde attenuates AS via inhibiting the I*κ*B/NF-*κ*B signaling pathway in a high fat diet-induced ApoE -/- mouse model [49]. Here, we focused our efforts at examining the effects of baicalin. This agent is a naturally occurring bioactive compound in S. baicalensis Georgi (SBG) which exerts prophylactic and/or therapeutic effects via regulating lipid metabolism, reducing inflammation-induced damage, inhibiting oxidative stress and altering immune regulation [50]. Due to these effects it has been reported to be a promising therapeutic agent for treating diabetes, cardiovascular or cerebrovascular disease, carcinogenesis as well as other diseases [51]. Results from previous studies have shown that baicalin exerts anti-inflammatory effects by inhibiting TLR4/NF-*κ*B signaling pathways [52, 53]. In our study, we present the first evidence that upregulation of IL-1*β* mRNA expression and increases in phosphorylated NF-*κ*B (p65) protein, as induced by thrombin, is significantly reduced by baicalin, thereby producing a protective effect on VSMC inflammation in AS. Baicalin also inhibited the thrombin-induced proliferation of VSMCs involved in AS. Moreover, relatively high concentrations of 10 to 50 uM baicalin failed to produce any cytotoxic effects in VSMCs. These findings, which demonstrate the effectiveness and safety of baicalin, suggest that it may be a promising therapeutic agent for AS. Further work will be required to identify the molecular mechanisms of baicalin which remain unclear.

To investigate the possible mechanism through which baicalin pretreatment inhibited this thrombin-induced inflammatory effect upon VSMCs, we examined the effects of baicalin on the thrombin-induced expression of PAR-1. In our study, we found that an administration of baicalin inhibited the thrombin-induced upregulation of PAR-1 mRNA and protein, suggesting that the anti-inflammatory effect of baicalin on VSMCs exposed to thrombin may, in part, be mediated by suppression of PAR-1 upregulation [23]. Among several signaling pathways regulating the inflammation process within VSMCs in AS, MAPK pathways play a key role, with the ERK1/2 kinase considered as a vital signaling pathway involved in thrombin-induced cell inflammation and proliferation mediated by PAR-1 [11, 54]. Here, our findings revealed that thrombin-induced inflammation due to an upregulation in the expression of PAR-1 in VSMCs appeared to be mediated by ERK1/2 activation, evidenced by increased ERK1/2 phosphorylation, while administration of baicalin attenuated this increased phosphorylation of ERK1/2. Taken together, our current results suggest that baicalin could inhibit the thrombin-induced activation of ERK1/2 signaling in VSMCs and thus exert a protective effect against inflammation as mediated by a thrombin-induced upregulation of PAR-1 in AS.

## 5. Conclusion

In conclusion, our study showed that thrombin could induce VSMC inflammation resulting in the pathogenesis of AS by upregulating the expression of PAR-1. Importantly, baicalin could produce a protective effect against VSMC inflammation mediated by thrombin-induced upregulation of PAR-1, which may be mediated by its inhibitory effects upon the thrombin-induced activation of the ERK1/2 pathway. Baicalin, a traditional Chinese drug, may be a safe and promising candidate for the treatment of AS.

## Figures and Tables

**Figure 1:** Thrombin induces proliferation of VSMCs. Cell viability was examined by CCK-8 assay in VSMCs. Cells were treated with various doses of thrombin for 24 h (a) and 2.5 U/ml thrombin for various times (b). ^∗^*p* < 0.05,^∗∗^ *p* < 0.01, and ^∗∗∗^*p* < 0.005.

**Figure 2:** Thrombin induces inflammation in VSMCs. (a) The expression of IL-1*β* mRNA in VSMCs treated with different doses of thrombin was determined by RT-PCR. (b) Western blot analysis of p-P65 and P65 protein expression in VSMCs treated with thrombin and quantification.^∗^*p* < 0.05,^∗∗^ *p* < 0.01, and ^∗∗∗^*p* < 0.005.

**Figure 3:** Thrombin induces upregulation of PAR-1 in VSMCs. (a) The expression of PAR-1 mRNA in VSMCs treated with different doses of thrombin was measured by RT-PCR. (b) Western blot analysis and quantification of PAR-1 protein expression in VSMCs treated with thrombin. ^∗^*p* < 0.05,^∗∗^ *p* < 0.01, and ^∗∗∗^*p* < 0.005.

**Figure 4:** Baicalin inhibits thrombin-induced proliferation of VSMCs. CCK-8 assay of cell viability of VSMCs treated with (a) 2.5 U/ml thrombin with various doses of baicalin or (b) various doses of baicalin for 24 h.^∗^*p* < 0.05,^∗∗^ *p* < 0.01, and ^∗∗∗^*p* < 0.005.

**Figure 5:** Baicalin alleviates thrombin-induced inflammation in VSMCs. (a) The expression of IL-1*β* mRNA in VSMCs after exposure to 2.5 U/ml thrombin pre-treated with or without baicalin was determined by RT-PCR. (b) Western blot analysis and quantification of the protein level of p-P65 and P65 in VSMCs stimulated by 2.5 U/ml thrombin after pretreatment with different doses of baicalin.^∗^*p* < 0.05,^∗∗^ *p* < 0.01, and ^∗∗∗^*p* < 0.005.

**Figure 6:** Baicalin inhibits VSMC inflammation by suppressing thrombin-induced PAR-1 expression. (a) The expression of PAR-1 mRNA in VSMCs after exposure to 2.5 U/ml thrombin pre-treated with or without baicalin was determined by RT-PCR. (b) Western blot analysis and quantification of PAR-1 protein level in VSMCs stimulated by 2.5 U/ml thrombin after pretreatment with different doses of baicalin. (c) Immunofluorescence microscopy of punctate pattern of PAR-1 localization in VSMCs treated with 2.5 U/ml thrombin with or without baicalin.^∗^*p* < 0.05,^∗∗^ *p* < 0.01, and ^∗∗∗^*p* < 0.005.

**Figure 7:** The inhibitory effect of baicalin on VSMC inflammation induced by thrombin-PAR-1 is mediated via ERK1/2 signaling. (a) After exposure to different doses of thrombin, the level of phosphorylated ERK1/2 was evaluated by western blot analysis. (b) Western blot analysis and quantification of phosphorylated ERK1/2 protein level after exposure to 2.5 U/ml thrombin with or without baicalin.^∗^*p* < 0.05,^∗∗^ *p* < 0.01, and ^∗∗∗^*p* < 0.005.

## Data Availability

The data used during this study are available from the corresponding author on reasonable request.
